# An Improved Ant Colony Optimization Approach for Optimization of Process Planning

This article has been retracted.

**DOI:** 10.1155/2014/294513

**Published:** 2014-07-06

**Authors:** JinFeng Wang, XiaoLiang Fan, Haimin Ding

**Affiliations:** School of Energy, Power and Mechanical Engineering, North China Electric Power University, Baoding 071003, China

## Abstract

Computer-aided process planning (CAPP) is an important interface between computer-aided design (CAD) and computer-aided manufacturing (CAM) in computer-integrated manufacturing environments (CIMs). In this paper, process planning problem is described based on a weighted graph, and an ant colony optimization (ACO) approach is improved to deal with it effectively. The weighted graph consists of nodes, directed arcs, and undirected arcs, which denote operations, precedence constraints among operation, and the possible visited path among operations, respectively. Ant colony goes through the necessary nodes on the graph to achieve the optimal solution with the objective of minimizing total production costs (TPCs). A pheromone updating strategy proposed in this paper is incorporated in the standard ACO, which includes Global Update Rule and Local Update Rule. A simple method by controlling the repeated number of the same process plans is designed to avoid the local convergence. A case has been carried out to study the influence of various parameters of ACO on the system performance. Extensive comparative experiments have been carried out to validate the feasibility and efficiency of the proposed approach.

## 1. Introduction

Process planning for prismatic parts is a very complex and difficult process. For a prismatic part with complex structures and numerous features, process planning involves selecting machining operations for every feature and sequencing them considering precedence constraints, choosing available manufacturing resources, determining setup plans, and machining parameters, and so forth. In CAPP systems, these activities can be carried out simultaneously to achieve an optimal plan, thus the manufacturing efficiency could be largely increased or the production cost could be decreased. So, process planning problem is well known as a combinatorial optimization problem with constraints. With the advance of computer technology, some artificial intelligence (AI) techniques are used to solve combinatorial optimization problem. For example, some bioinspired algorithms are applied in complex decision-making process of solve combinatorial optimization problem [1–3].

In this paper, an improved ant colony optimization (ACO) approach is proposed to deal with process planning problem based on a weight graph. The weighted graph consists of nodes, directed arcs, and undirected arcs, which denote operations, precedence constraints among operation, and the possible visited path among operations, respectively. Ant colony goes through the operation nodes on the graph along the directed/undirected arcs. The heuristic information of operation nodes and pheromone amount on the arcs will guide ant colony to achieve the optimal nodes set and arc set, which represents the optimal solution with the objective of minimizing total production costs (TPCs). Some efforts have been adopted to improve the efficiency of the approach.

## 2. Previous Related Works

In the past two decades, CAPP has received much attention [4–7]. Many optimization approaches have been developed and widely applied for solving process planning problem, such as knowledge-based reasoning approach [8, 9], genetic algorithm (GA) [1, 5, 10], artificial neural networks (ANN) [11], graph manipulation [7, 12], tabu search approach (TS) [6, 13], simulated annealing algorithm (SA) [13, 14], artificial immune system (AIS) [15], particle swarm optimization (PSO) [16, 17], and ant colony optimization (ACO) [18, 19].

Zhang et al. [5] constructed a novel computer-aided process planning model consisting of operation selecting and operation sequencing. A GA is proposed for process planning based on the model considering a job shop manufacturing environment. GA is used to select machining resources and sequence operations simultaneously. Ma et al. [14] modeled the constraints of process planning problems in a concurrent manner. Precedence relationships among all the operations are used to generate the entire solution space with multiple planning tasks. Based on the proposed model, an algorithm based on simulated annealing (SA) is proposed to search for the optimal solution. Li et al. [6] consider the process planning problem as a constraint-based optimization problem and propose a tabu search-based algorithm to solve it. In the proposed algorithm, costs of the machines and tools, machine changes, tool changes, setups, and penalty against good manufacturing practices are taken as the evaluation criteria. Precedence constraints between features and the corresponding operations are defined and classified according to their effects on the plan feasibility and processing quality. Chan et al. [15] model the machine tool selection and operation allocation of flexible manufacturing systems and solve process problem by a fuzzy goal—programming approach based on artificial immune systems. Guo et al. [16] proposed a PSO approach for process planning problem. The initial process plans randomly generated are encoded into particles of the PSO algorithm. To avoid falling into local optimal and improve moving efficient of the particles, several new operators have been developed. Penalty strategy is used considering the evaluation of infeasible particles. Krishna and Mallikarjuna Rao [18] proposed a novel approach to apply the ant colony algorithm as a global search technique for process planning problem by considering various feasibility constraints.

Recently, to improve the quality of results and efficiency of the search, many hybrid approaches are developed for process planning problem, for example, GA + SA [13], graph manipulation + GA [7], and local search algorithm + PSO [20]. Li et al. [6] developed a hybrid genetic algorithm and a simulated annealing approach for optimizing process plans for prismatic parts. They modeled the process planning as a combinatorial optimization problem with constraints. The evaluation criterion was the combination of machine costs, cutting tool costs, machine change costs, tool change, and setup costs. Ding et al. [20] proposed a hybrid approach to incorporate a genetic algorithm, neural network, and analytical hierarchical process (AHP) for process planning problem. A globally optimized fitness function is defined including the evaluation of manufacturing rules using AHP, calculation of cost and time, and determination of relative weights using neural network techniques. Huang et al. [7] model the process planning problem as a combinatorial optimization problem with constraints and developed a hybrid graph and genetic algorithm (GA) approach. In the approach, graph theory accompanied with matrix theory is embedded into the main frame of GA. The precedence constraints between operations are formulated in an operation precedence graph (OPG). An improved GA was applied to solve process planning problem based on the operation precedence graph (OPG). Wang et al. [21] proposed an optimization approach based on particle swarm optimization (PSO) to solve the process planning problem and introduced a novel solution representation scheme for the application of PSO. In the hybrid approach, two kinds of local search algorithms are incorporated and interweaved with PSO evolution to improve the best solution in each generation.

Although significant improvements have been achieved for process planning problem, there still remains potential for further improvement [22]. For example, optimization approach needs to be improved to be more efficient, and a more reasonable constraint modeling and handling mechanism needs to be developed; also, some practical manufacturing environment should be considered, and the approach should provide the multiple alternative optimal plans. Especially, some bioinspired algorithms are improved to solve the complicated combination optimization problem [23, 24]. The attempt to use these algorithms to solve process planning problem should be performed to explore the more excellent results.

## 3. Graph-Based Process Planning Problem

In CAPP, a part is generally described by manufacturing features, which are geometric forms having machining meanings, such as holes, slots, and bosses. In the process planning for the part, the manufacturing features will be recognized by analyzing the geometrical and topological information of the part, which include position, dimensions, tolerance, and surface finish. A feature may be mapped to one or several sets of operation types (OPTs) [5]. An OPT refers to an operation without any attachment of machine (*M*), tool (*T*), and tool approach direction (TAD).

For an operation, there are a set of Ms, Ts, and TADs under which the operation can be executed. As a result, for a part, the process plan is a set of operations, which is represented as follows:

(1) $$\begin{array}{c} \text{PP}=\left\{{\text{OP}}_{1},{\text{OP}}_{2},\ldots ,{\text{OP}}_{i}\right\}, \end{array}$$

where OP_*i*_ is the *i*th operation of the part, which is defined as follows:

(2) $$\begin{array}{c} {\text{OP}}_{i}=\left\{{\text{OPT}}_{i1},{\text{OPT}}_{i2},\ldots ,{\text{OPT}}_{ij},\ldots ,{\text{OPT}}_{in}\right\}, \end{array}$$

where OPT_*ij*_ is the *j*th alternative operation of the *i*th operation of the part, which is defined as follows:

(3) $$\begin{array}{c} {\text{OPT}}_{ij}=\left\{M_{ij},T_{ij},{\text{TAD}}_{ij}\right\}, \end{array}$$

where *M*_*ij*_, *T*_*ij*_, and TAD_*ij*_ are the index of the machine, tool, and TAD respectively, by which the alternative operation OPT_*ij*_ is executed.

In process planning for a part, two tasks have to be done, namely, selecting operation OP_*i*_ for each feature of the part and sequencing operations. And, also, they must be carried out simultaneously to achieve an optimal process plan against a predetermined criterion. Due to the geometrical and manufacturing constraints between manufacturing features, operation sequencing must take into account the precedence constraints between operations, which must be satisfied by the final operations sequence. Many constraints and rules have been proposed and summarized [1, 5, 7]. In general, these precedence constraints are as follows [19]:

1. primary surfaces prior to secondary surfaces,
2. planes prior to its associated features,
3. rough machining operation prior to finish machining operation,
4. datum surfaces prior to its associated features, and
5. some good manufacturing practice.

To construct process plan with the ACO approach, the process planning problem has to be visualized and represented by a weighted graph. The weighted graph is denoted as *D* = (*O*, *C*, *U*), where *O* is a set of nodes, *C* is a set of directed arcs, and *U* is a set of undirected arcs. The nodes of *O* stand for all of the operations OP_*i*_. *C* corresponds to the precedence constraints between the operations of the parts. *U* represents the set of arcs connecting all possible combinations of the nodes. Both *C* and *U* represent possible paths for ants travelling from one node to another. The ants are basically free to travel along the paths unless there is a precedence constraint specified by *C*. In this paper, an example part is used to illustrate the weighted graph [2].

The alternative operations for the example in Figure 1 are listed in Table 1. The precedence constraints for the example are listed in Table 2.

Figure 2 is the weighted graph for the example part. The set of nodes includes five nodes, *O*_1_, *O*_2_, *O*_3_, *O*_4_, and *O*_5_, which represent the operations OP_1_, OP_2_, OP_3_, OP_4_, and OP_5_. The set of directed arcs includes four arcs, *C*_1_, *C*_2_, *C*_3_, and *C*_4_, which represent the precedence constraints 1, 2, 3, and 4. The set of undirected arcs includes six arcs, *U*_1_, *U*_2_, *U*_3_, *U*_4_, *U*_5_, and *U*_6_.

While applying the ACO in the process planning by the weighted graph, the ant colony will be placed on the initial node visited by the ant colony first. The initial node determines which operation can be executed first. For the weighted graph in Figure 2, the nodes *O*_1_ and *O*_5_ are likely to be selected as the initial source node, since operations OP_1_ and OP_5_ have no precedence operations. To facilitate the execution of ACO in process planning, a dummy node *O*_*b*_ acting as the initial node is added to connect the possibly executed operations first in the weighted graph. The initial node *O*_*b*_ is used to connect the nodes *O*_1_ and *O*_5_.

## 4. Process Plan Evaluation Criterion

Lots of process planning evaluation criteria have been proposed in the past literatures. The criterion of minimum production cost is generally used. The production cost evaluating process plans comprise five factors: machine processing cost (MC), tool processing cost (TC), machine change cost (MCC), tool change cost (TCC), and set-up change cost (SCC) [6, 8, 9, 12, 13]. The calculation procedures of these cost factors are described in detail below:

(1) total machine cost (TMC):
  (4) $$\begin{array}{c} \text{TMC}=\overset{n}{\underset{i=1}{\sum }}{\text{MC}}_{i}, \end{array}$$
 where *n* is the total number of operations and MC_*i*_ is the machine cost of the *i*th machine for an operation, a constant for a specific machine;
(2) total tool cost (TTC):
  (5) $$\begin{array}{c} \text{TTC}=\overset{n}{\underset{i=1}{\sum }}{\text{TC}}_{i}, \end{array}$$
 where TC_*i*_ is the tool cost of the *i*th tool for an operation, a constant for a specific machine;
(3) total setup cost (TSC):
  (6) $$\begin{array}{c} \text{TSC}=\text{SCC}*\text{NS}, \end{array}$$
 where SCC is the setup cost and NS is the number of setups, which can be calculated by
  (7) $$\begin{array}{c} \text{NS}=\text{NSC}+1,\\ \text{NSC}=\overset{n-1}{\underset{i=1}{\sum }}\Omega_{2}\left(\Omega_{1}\left(M_{i+1},M_{i}\right),\Omega_{1}\left({\text{TAD}}_{i+1},{{\text{TAD}}_{i}}_{i}\right)\right), \end{array}$$
 where TAD_*i*_ is the *i*th TAD;
(4) total machine change cost (TMCC):
  (8) $$\begin{array}{c} \text{TMCC}=\text{MCC}*\text{NMC}, \end{array}$$
 where MCC is machine change cost and NMC is number of machine change, which can be calculated by
  (9) $$\begin{array}{c} \text{NMC}=\overset{n-1}{\underset{i=1}{\sum }}\Omega_{1}\left(M_{i+1},M_{i}\right), \end{array}$$
  (10) $$\begin{array}{c} \Omega_{1}\left(x,y\right)=\{\begin{array}{cc} 1 & x\neq y\\ 0 & x=y, \end{array} \end{array}$$
 where *M*_*i*_ is the machine for the *i*th operation;
(5) total tool change cost (TTCC):
  (11) $$\begin{array}{c} \text{TTCC}=\text{TCC}*\text{NTC}, \end{array}$$
 where TCC is the tool change cost and NTC is the number of tool change, which can be calculated by (10) and
  (12) $$\begin{array}{c} \text{NTC}=\overset{n-1}{\underset{i=1}{\sum }}\Omega_{2}\left(\Omega_{1}\left(M_{i+1},M_{i}\right),\Omega_{1}\left(T_{i+1},T_{i}\right)\right), \end{array}$$
  (13) $$\begin{array}{c} \Omega_{2}\left(x,y\right)=\{\begin{array}{cc} 0 & x=y=0\\ 1 & \text{otherwise}, \end{array} \end{array}$$
 where *T*_*i*_ is the *i*th tool.

The definition of machine change, tool change, and setup change has been illustrated in detail [6, 9]. In this paper, the combination of TWC, TTC, TMCC, TTCC, and TSCC will be used as the objective of process planning problem, which can be defined as total production cost (TPC) andcalculated by

(14) TPC=w1∗TMC+w2∗TTC+w3∗TMCC+w4∗TTCC+w5∗TSCC.

In (14), *w*_1_, *w*_2_, *w*_3_, *w*_4_, and *w*_5_ are weights of TMC, TTC, TMCC, TTCC, and TSCC, respectively, the value of which is limited in {0,1}. These weights can be assigned referring to the active situations, which provides the flexibility to customize the optimization objective function according to various situations [13].

## 5. The Proposed ACO Algorithm

The proposed ACO algorithm basically generates solutions by standard ACO procedures [2]. As described in Section 3, the directed graphs are used to represent the process planning problem [19, 25]. The approach in this paper is to solve the process planning problems using the ACO algorithm which corresponds to finding a path of the directed graph, where all necessary nodes have to be visited to complete the process plan, so that the objective of process planning is minimized. The explanations for symbols used are listed in the Symbols section.

### 5.1. Heuristic Information

To choose the next visiting node, the ant *k* is guided by the heuristic information *η*_*uv*_ on the node and the pheromone amount *τ*_*uv*_ on the arc linking the source node *u* and possible destination node *v*. *η*_*uv*_ is defined simply by a greedy heuristic

(15) $$\begin{array}{c} \eta_{uv}=\frac{E}{\text{PC}}, \end{array}$$

where *E* is a positive constant, and it can be set by trial and error. Therefore, the nodes with the smaller processing cost have the higher heuristic information amount and these nodes have more attraction for the ant *k*. PC is the processing cost of the selected node operation and it is calculated as follows:

(16) $$\begin{array}{c} \text{PC}=w_{1}*{\text{MC}}_{i}+w_{2}*{\text{TC}}_{i}. \end{array}$$

MC_*i*_ is illustrated in (4). TC_*i*_ is illustrated in (5). *w*_1_ and *w*_2_ are illustrated in (14).

### 5.2. Selection Probability

The heuristic information and the pheromone amount constructed a probability of moving from a node to another node for an ant. The more the pheromone amount on the arcs and the heuristic information on the nodes, the higher the selective probability. For the ant *k*, the selective probability *p*_*uv*_^*k*^ from the source node *u* to the destination node *v* can be given as follows:

(17) $$\begin{array}{c} p_{uv}^{k}=\{\begin{array}{cc} \frac{{\left[\tau_{uv}^{k}\right]}^{\alpha }{\left[\eta_{uv}\right]}^{\beta }}{\sum_{w\in S_{k}}{\left[\tau_{uw}^{k}\right]}^{\alpha }{\left[\eta_{uv}\right]}^{\beta }} & v\in S_{k}\\ 0 & v\notin S_{k}, \end{array} \end{array}$$

where *α* and *β* denote the weighting parameters controlling the relative importance of the pheromone amount and the heuristic information, respectively. *S*_*k*_ is the set of nodes allowed at the next step for the ant *k*.

In order to adjust the convergence speed of the algorithm, a simple pheromone updating strategy is proposed in the standard ACO, which includes two pheromone updating rules. Local Update Ruler for the elite process plan is incorporated into Global Update Ruler. Three types of process planning solutions are specified at different stages of the algorithm so as to incorporate the pheromone updating strategy. Iteration best process plan PP_*i*_ denotes the best process plan generated in the current iteration by the total number of ants *K*, whose TPC is *L*_*i*_. Restart best process plan PP_*r*_ denotes the best process plan generated since the last restart of the algorithm, whose TPC is *L*_*r*_. Algorithm best process plan PP_*b*_ denotes the best process plan generated since the start of the algorithm, whose TPC is *L*_*b*_. *L*_avg_ is the average TPC since the restart of the algorithm and is calculated as follows:

(18) $$\begin{array}{c} L_{\text{avg}}=\frac{\sum_{i=1}^{R_{\text{ite}}}L_{i}}{R_{\text{ite}}}. \end{array}$$

### 5.3. Global Update Ruler

The pheromone level is initially set at *τ*_0_ on every arc. Pheromone intensity on the arcs is dynamically updated after ant colony has completed process plans. The amount of pheromone deposited on the arcs by an ant *k* is proportional to respective *L*_*k*_. The process plans with smaller *L*_*k*_ will accumulate a greater amount of pheromone on their corresponding arcs. To avoid unlimited accumulation of the pheromone, the pheromone also evaporates at every round of iterations. The pheromone amount *τ*_*uv*_ can be given as follows:

(19) $$\begin{array}{c} \tau_{uv}^{k}=\left(1-\rho \right)*\tau_{uv}^{k}+\Delta \tau_{uv}^{k}, \end{array}$$

where *ρ* is an evaporation coefficient of the pheromone on the arc linking the source node *u* and possible destination node *v*. Δ*τ*_*uv*_^*k*^ is the quantity of the pheromone increments on the arc(*u*, *v*) generated by the ant *k* after each iteration. Also, it can be given as

(20) $$\begin{array}{c} \Delta \tau_{uv}^{k}=\{\begin{array}{cc} \frac{Q}{L_{k}} & \text{if}\;L_{k}\leq L_{\text{avg}}\;\text{ant}\;k\;\text{passes}\;\text{the}\;\text{arc}\left(u,v\right)\\ 0 & \text{otherwise}, \end{array} \end{array}$$

where *Q* is a positive constant. *L*_*k*_ is the TPC by the ant *k*.

### 5.4. Local Update Rule

Local Update Rule is introduced so that the elite process plan solutions are used to update the pheromone on the arcs again, which will accelerate the convergence of the algorithm to the optimal process plan. The iteration best process plan PP_*i*_ is first identified from all the ant process plans PP_*k*_. If the *L*_*i*_ is smaller than that of *L*_*r*_, *L*_*r*_ is replaced by *L*_*i*_. Similarly, if *L*_*r*_ is smaller than that of *L*_*b*_, *L*_*b*_ is replaced by *L*_*r*_. Local Update Rule is used to update the pheromone intensity on the arcs again while update of *L*_*r*_ and *L*_*b*_ occurs.The pheromone amount *τ*_*uv*_ can be calculated as (19), and Δ*τ*_*uv*_^*k*^ will be calculated as follows:

(21) Δτuvk={QLkif (Lk≤Lr  or  Lk≤Lb) ant k passes the arc(u,v)0otherwise,

where *Q* is a positive constant. *L*_*k*_ is the TPC by the ant *k*.

### 5.5. Termination

If all of the ants almost constructed the same process plan repeatedly at the early stage of the ACO algorithm, the algorithm would fall into the local convergence, which leads to failure in the exploration of new paths for the subsequent iteration. This is derived from an extraordinary accumulation of pheromone placed on the same set of arcs visited by the ants. Once the algorithm has fallen into the local convergence, the output of process planning would not be the optimal result, even far from the optimal results. To void the local convergence, the parameter of *M*_rpt_ controlling the repeated number of the same process plan is set in advance. When the adjacent two process plans are completely the same, the variable of *N*_rpt_ will increase by 1; otherwise *N*_rpt_ will be reset to be 0. When *N*_rpt_ reaches *M*_rpt_, it means that no improvement on the solutions is made in the recent iterations. The ants may have converged to local optimal results. If the two events of *N*_rpt_ = *M*_rpt_ and *N*_ite_ < *M*_ite_ are satisfied simultaneously, it is considered that the local convergence occurs and the algorithm will be restarted. For the case where the algorithm is restarted, all the pheromones are reset to their initial value *τ*_0_, *R*_ite_ isreset to be 0, and *L*_*r*_ is reinitialized. In this case, the ants are able to escape from one particular solution to other possible paths and hence the search space will be increased. If the only event of *N*_ite_ = *M*_ite_ is satisfied, the resulting process plan will be output and algorithm will be terminated.

## 6. Experiments and Results

Two experiments have been conducted to illustrate and validate the feasibility and efficiency of the proposed approach. In the first experiment and the crucial parameters of the approach are determined. The second experiment is used to compare this approach with typical ACO, TS, GA, and SA methods.

Two prismatic parts are used for the case experiments. The first prismatic part (Part 1) used by Zhang et al. [5] is illustrated in Figure 3. It consists of 14 STEP-defined manufacturing features and 14 machining operations. The machining information and precedence constraints are given in Tables 3 and 4. The second prismatic part (Part 2) used by Li et al. [13] is illustrated in Figure 4. The machining information and precedence constraints are given in Tables 5 and 6.

### 6.1. Simulation Experiments

When ACO is applied in process planning, those parameters including *K*, *ρ*, *α*, *β*, *E*, *Q*, *τ*_0_, *M*_ite_, and *M*_rpt_ have to be adjusted according the situation to achieve the optimal process plan. A lot of preliminary experiments are dominated to test the effect of various parameters. In each experiment, one parameter is changed and the other parameters are fixed, and the effect of the changed parameter on the algorithm properties was analyzed at different levels. The process planning problem for Part 1 is used to illustrate how the crucial parameters are determined. It is assumed that all the machines and tools are available; namely, *w*_1_–*w*_5_ in (14) and (16) are set as 1.

Those parameters may be analyzed from three aspects, namely, initial parameters of ACO (*K*, *ρ*, *α*, *β*, and *τ*_0_), problem data (*M*_ite_ and *M*_rpt_), and problem size (*E*, *Q*). Firstly, the positive constants *E* and *Q* in (15), (20), and (21) are determined according to problem size, which includes average PC of each operation node and average TPC of process plan appearing in the previous paper. For Part 1, while the initial pheromone intensity on all the arcs *τ*_0_ is set to 1, *E* and *Q* are fixed at 50 and 2000, respectively. Secondly, since an updating strategy including two updating rules is applied in the proposed ACO, the maximum iteration number *M*_ite_ just needs to guarantee the algorithm convergence. The maximum repeat number *M*_rpt_ affects the performance of ACO and optimization result.

Thirdly, initial parameters of ACO algorithm affect the performance of process planning using ACO. The effect is described and illustrated by an analysis of the application of the proposed ACO algorithm in the process planning problem for Part 1. Number of ants *K* has important effect on the convergence speed. If *K* is too small, searching randomness of ACO will increase and the computation time will be long. If *K* is too large, the optimization rate will become very slow. Generally, value of *K* is considered according to the problem size. In the case of problems with *ρ* = 0.75, *α* = 1, *β* = 1, *τ*_0_ = 1, *E* = 50, *Q* = 2000, *M*_ite_ = 300, and *M*_rpt_ = 5, 10 trials were separately conducted by varying the values of *K* ∈ {10,25,40}. The average results of the experiment are summarized in Figure 5.

All the hills and troughs on the TPC of *L*_*i*_ and *L*_*r*_ in Figures 5(a) and 5(b) denote the restart of the algorithm. They indicate that the local convergence avoidance mechanism takes effect to direct the ants from one solution region to another.  Figure 5(b) shows that there are 10, 7, and 5 restarts corresponding to *K* = 10, *K* = 25, and *K* = 40 within the 300 iterations.  Figure 5(c) shows that the compared results under *K* = 10, *K* = 25, and *K* = 40. Accordingly, *K* was determined as 25.

A suitable *ρ* can ensure good computational efficiency and algorithm stability. In the case of problems with *K* = 25, *α* = 1, *β* = 1, *τ*_0_ = 1, *E* = 50, *Q* = 2000, *M*_ite_ = 300, and *M*_rpt_ = 5, 10 trials were separately conducted by varying the values of *ρ* ∈ {0.25,0.5,0.75}. The average results of *L*_*b*_ achieved by the algorithm best process PP_*b*_ are summarized in Figure 6.

In the case of problems with *K* = 25, *ρ* = 0.75, *τ*_0_ = 1, *E* = 50, *Q* = 2000, *M*_ite_ = 300, and *M*_rpt_ = 5, 10 trials were separately conducted by varying the values of *α* ∈ {0.1,1, 5} and *β* ∈ {0.1,1, 5}. The average results of *L*_*r*_ achieved by the restart best process PP_*r*_ are summarized in Table 7.

50 trials were separately conducted to evaluate the performance of the proposed approach. The results show that these parameters have a good performance at values *K* = 25, *ρ* = 0.75, *α* = 1, *β* = 1, *τ*_0_ = 1, *E* = 50, *Q* = 2000, *M*_ite_ = 300, and *M*_rpt_ = 5, under which one of the best process plans is shown in Table 8 and the corresponding simulation results of *L*_*r*_ and *L*_*b*_ are in Figure 7.

Figure 7 shows that there are 7 restarts within the 300 iterations. When iterations are between 34 and 38, the ants repeatedly generate plans without any further improvement on the TPC under 1143. The local convergence avoidance mechanism is triggered to renew all the pheromone trails and bring the ants to other search regions. Therefore, the first restart occurs on the iteration 39, on which the ants are released to construct process plans with a TPC of 1348. Although it is larger than 1143, the ACO algorithm is able to bring the ants to the better solutions again.

The above experiments are based on Part 1. To ensure that these parameters are applicable in other situations, the extensive comparative experiments for Part 2 will use the same chosen parameters.

### 6.2. Extensive Comparative Experiments

Three conditions are used to test proposed algorithm for the sample parts [6, 13].

1. All machines and tools are available, and *w*_1_–*w*_5_ in (11) and (13) are set as 1.
2. All machines and tools are available, and *w*_2_ = *w*_5_ = 0; *w*_1_ = *w*_3_ = *w*_4_ = 1.
3. Machine M2 and tool T7 are down, and *w*_2_ = *w*_5_ = 0; *w*_1_ = *w*_3_ = *w*_4_ = 1.

Under condition (1), condition (2), and condition (3), 10 trials were separately conducted to evaluate the proposed algorithm's performance for Part 2. Experimental observation has shown that *K* = 40, *ρ* = 0.75, *α* = 2, *β* = 1, *τ*_0_ = 1, *E* = 100, *Q* = 3000, *M*_ite_ = 300, and *M*_rpt_ = 5 are the best choices of these parameters. Under condition (1), one of the best operation sequences is shown in Table 9. Under condition (2), one of the best operation sequences is shown in Table 10. Under condition (3), one of the best operation sequences using proposed algorithm is shown in Table 11.

In Table 12, the TPCs generated by the proposed ACO are compared with those of GA and SA approach by Li et al. [13], TS by Li et al. [6], and the ACO by Liu et al. [19]

The comparing results show that the proposed algorithm is better than the other algorithms. Under condition (1), a lower TPC (2435.0) has been found using the improved ACO approach, and the mean TPC (2456.1) is better than the costs of other four algorithms. Under condition (2), a lower TPC (1970.0) has been found using the improved ACO approach. Under condition (3), the minimum TPC (2580) is the same as the TS [6]. The mean TPC generated by proposed approach is better than the other algorithms under the three conditions.

## 7. Conclusions

An improved ACO approach is developed to solve the process planning optimization problem for prismatic parts. The approach is characterized by the following aspects.

1. A weighted graph is used to represent process planning problem. The graph includes nodes set, directed arcs set, and undirected arcs set, which denote operations, precedence constraints between the operations, and possible visited path connecting the nodes, respectively.
2. A pheromone updating strategy proposed in the proposed ACO is incorporated in the standard ACO, which includes Global Update Rule and Local Update Rule. A simple method by controlling the repeated number of the same process plan is designed to avoid the local convergence.

In a further study, a deep discussion of selecting the ACO approach parameters is conducted. In addition, the multiobjective optimization will be incorporated into the ACO approach for handling the multiobjective process planning problem.

## Figures and Tables

**Figure 1:** An example part [5].

**Figure 2:** Weighted graph for the example part.

**Figure 3:** A sample part with 14 features and 14 operations: Part 1.

**Figure 4:** A sample part with 14 features and 20 operations: Part 2.

**Figure 5:** Determination of numbers of ants *K*.

**Figure 6:** Determination of pheromone evaporation rate *ρ*.

**Figure 7:** Simulation results of *L*_*r*_ and *L*_*b*_ corresponding to one of the best process plans.

**Table 1:** Operation selection for the example part.

Feathers	Operations	Machines	Tools	TADs	Description
F1	Drilling (OP_1_)	M1	T1	−*Y*	M1: Vertical milling center
		M2	T1		M2: Drill press
F2	Milling (OP_2_)	M1	T2	+*Z*	T1: Drill
F3	Milling (OP_3_)	M1	T4	−*Z*	T2: End mill
			T5	−*Z*	T3 Drill
			T4	+*Y*	T4: Chamfer cutter
			T5	+*Y*	T5: Ball-nose cutter
F4	Drilling (OP_4_)	M1	T3	−*Z*	T6: T-slot cutter
		M2			
F5	Milling (OP_5_)	M1	T2	+*Z*	
			T6	+*Y*	

**Table 2:** Precedence constraints for the example part.

ID	Features	Operations	Precedence constraints description
1	F1	OP_1_	*CO*_1_ is prior to *CO*_2_
2	F2	OP_2_	*CO*_2_ is prior to *CO*_4_
3	F4	OP_4_	*CO*_4_ is prior to *CO*_3_
4	F5	OP_5_	*CO*_5_ is prior to *CO*_3_

**Table 3:** Features, operations, and machining information for Part 1.

Features	Feature descriptions	Operations	TADs	Machines	Tools	Remarks
F1	Two replicated holes	Drilling (OP_1_)	+*Z*, −*Z*	M1, M2, M3	T1	M1(10):Drill press
F2	A chamfer	Milling (OP_2_)	−*X*, +*Y*, −*Y*, −*Z*	M2, M3	T8	M2(35):Vertical milling
F3	A slot	Milling (OP_3_)	+*Y*	M2, M3	T5, T6	M3(60):Vertical CNC milling
F4	A slot	Milling (OP_4_)	+*Y*	M2	T5, T6	T1(3):Drill 1
F5	A step	Milling (OP_5_)	+*Y*, −*Z*	M2, M3	T5, T6	T2(3):Drill 2
F6	Two replicated holes	Drilling (OP_6_)	+*Z*, − *Z*	M1, M2, M3	T2	T3(8):Reamer
F7	Four replicated holes	Drilling (OP_7_)	+*Z*, − *Z*	M1, M2, M3	T1	T4(15):Boring tool
F8	A slot	Milling (OP_8_)	+*X*	M2, M3	T5, T6	T5(10):Milling cutter 1
F9	Two replicated holes	Drilling (OP_9_)	−*Z*	M1, M2, M3	T1	T6(15):Milling cutter 2
F10	A slot	Milling (OP_10_)	−*Y*	M2, M3	T5, T6	T7(10):Chamfer tool
F11	A slot	Milling (OP_11_)	−*Y*	M2, M3	T5, T7	T8(10):Slot cutter
F12	Two replicated holes	Drilling (OP_12_)	+*Z*, − *Z*	M1, M2, M3	T1	MCC = 300
F13	A step	Milling (OP_13_)	−*X*, − *Y*	M2, M3	T5, T6	SCC = 120
F14	Two replicated holes	Drilling (OP_14_)	−*Y*	M1, M2, M3	T1	TCC = 15

**Table 4:** Precedence constraints for Part 1.

Constraints	Descriptions	Hard or soft
Tool interactions	OP_1_ should be prior to OP_2_.	Hard
Datum interactions	OP_6_ should be prior to OP_7_.	Hard
	OP_10_ should be prior to OP_11_.	
	OP_13_ should be prior to OP_14_.	
Thin-wall interactions	OP_9_ should be prior to OP_8_.	Soft
	OP_12_ should be prior to OP_10_.	
Material removal interactions	OP_8_ should be prior to OP_9_.	Soft
	OP_10_ should be prior to OP_12_.	
	OP_13_ should be prior to OP_14_.	
	OP_3_ should be prior to OP_4_.	

**Table 5:** Features, operations, and machining information for Part 2.

Features	Feature descriptions	Operations	TADs	Machines	Tools	Remarks
F1	Planar surface	Milling (OP_1_)	+*Z*	M2, M3	T6, T7, T8	M1(10): Drilling press
F2	Planar surface	Milling (OP_2_)	−*Z*	M2, M3	T6, T7, T8	M2(40): Three-axis vertical milling machine
F3	Two replicated pockets	Milling(OP_3_)	+*X*	M2, M3	T6, T7, T8	
F4	Four replicated holes	Drilling(OP_4_)	+*Z*, −*Z*	M1, M2, M3	T2	M3(100): CNC 3-axis vertical milling machine
F5	A step	Milling (OP_5_)	+*X*, −*Z*	M2, M3	T6, T7	
F6	A protrusion (rib)	Milling (OP_6_)	+*Y*, −*Z*	M2, M3	T7, T8	M4(60): Boring machine
F7	A boss	Milling (OP_7_)	−*a*	M2, M3	T7, T8	T1(7): Drill 1
F8	A compound hole	Drilling (OP_8_)	−*a*	M1, M2, M3	T2, T3, T4	T2(5): Drill 2
		Reaming (OP_9_)		M1, M2, M3	T9	T3(3): Drill 3
		Boring (OP_10_)		M2, M3	T10	T4(8): Drill 4
F9	A protrusion (rib)	Milling (OP_11_)	−*Y*, −*Z*	M2, M3	T7, T8	T5(7): Tapping tool
F10	A compound hole	Drilling (OP_12_)	−*Z*	M1, M2, M3	T2, T3, T4	T6(10): Mill 1
		Reaming (OP_13_)		M1, M2, M3	T9	T7(15): Mill 2
		Boring (OP_14_)		M3, M4	T10	T8(30): Mill 3
F11	Nine replicated holes	Drilling (OP_15_)	−*Z*	M1, M2, M3	T1	T9(15): Ream
		Tapping (OP_16_)		M1, M2, M3	T5	T10(20): Boring tool
F12	A pocket	Milling (OP_17_)	−*X*	M2, M3	T7, T8	MCC = 160
F13	A step	Milling (OP_18_)	−*X*, −*Z*	M2, M3	T6, T7	SCC = 100
F14	A compound hole	Reaming (OP_19_)	+*Z*	M1, M2, M3	T9	TCC = 20
		Boring (OP_20_)		M3, M4	T10	

**Table 6:** Precedence constraints for Part 2.

Features	Operation	Precedence constraints description	Hard or soft
F1	Milling (OP_1_)	F1 (OP_1_) is the datum and supporting face for the part; hence it is machined prior to all features and operations.	Hard
F2	Milling (OP_2_)	F2 (OP_1_) is prior to F10 (OP_12_, OP_13_, and OP_14_) and F11 (OP_15_, OP_16_) for the material removal interactions.	Hard
F5	Milling (OP_5_)	F5(OP_5_) is prior to F4 (OP_4_) and F7(OP_7_) for the datum interactions	Hard
F6	Milling (OP_6_)	F6 (OP_6_) is prior to F10 (OP_12_, OP_13_, and OP_14_) for the datum interaction.	Hard
F7	Milling (OP_7_)	F7 (OP_7_) is prior to F8 (OP_8_, OP_9_, and OP_10_) for the datum interactions.	Hard
F8	Drilling (OP_8_)	OP_8_ is prior to OP_9_ and OP_10_; OP_9_ is prior to OP_10_ for the fixed order of machining operations.	Hard
	Reaming (*OP*_9_)		
	Boring (OP_10_)		
F9	Milling (OP_11_)	F9 (OP_11_) is prior to F10 (OP_12_, OP_13_, and OP_14_) for the datum interaction	Hard
F10	Drilling (OP_12_)	OP_12_ is prior to OP_13_ and OP_14_; OP_13_ is prior to OP_14_ for the fixed order of machining operations. F10 (OP_12_, OP_13_, and OP_14_) is prior to F11 (OP_15_, OP_16_), and OP_12_ of F10 is prior to F14 (OP_19_, OP_20_) for the datum interaction.	Hard
	Reaming (OP_13_)		
	Boring (OP_14_)		
F11	Drilling (OP_15_)	OP_15_ is prior to OP_16_ for the fixed order of operations.	Hard
	Tapping (OP_16_)		
F13	Milling (OP_18_)	F13 (OP_18_) is prior to F4 (OP_4_) and F12 (OP_17_) for the material removal interaction.	Soft
F14	Reaming (OP_19_)	OP_19_ is prior to OP_20_ for the fixed order of machining operations.	Hard
	Boring (OP_20_)		

**Table 7:** Determination of varying combinations of *α* and *β.*

	*α* = 0.1			α = 1			α = 5		
	β = 0.1	β = 1	β = 5	β = 0.1	β = 1	β = 5	β = 0.1	β = 1	β = 5
Mean	1137.1	1134.4	1132.6	1136.1	1129.1	1132.8	1336.6	1129.9	1136.9
Maximum	1150.5	1147	1143.5	1148.5	1137	1145	1149	1141.5	1149
Minimum	1131	1128	1128	1128	1128	1128	1128	1128	1129.5

**Table 8:** One of the best process plans for Part 1.

Operation	6	1	7	9	12	5	3	4	8	10	11	13	14	2
Machine	2	2	2	2	2	2	2	2	2	2	2	2	2	2
Tool	2	1	1	1	1	5	5	5	5	5	5	5	1	8
TAD	−*Z*	−*Z*	−*Z*	−*Z*	−*Z*	−*Z*	+*Y*	+*Y*	+*X*	−*Y*	−*Y*	−*Y*	−*Y*	−*Y*
NMC = 0, NTC = 4, NSC = 3, TMCC = 0, TTCC = 60, TSCC = 480, TMC = 490, TTC = 98, and TPC = 1128														

**Table 9:** One of the best process plans for Part 2 under condition (1).

Operation	1	2	18	11	6	12	13	19	17	3	5	7	8	9	10	20	14	4	15	16
Machine	2	2	2	2	2	2	2	2	2	2	2	2	2	2	2	4	4	1	1	1
Tool	7	7	7	7	7	3	9	9	7	7	7	7	3	9	10	10	10	2	1	5
TAD	+*Z*	−*Z*	−*Z*	−*Z*	−*Z*	−*Z*	−*Z*	+*Z*	−*X*	+*X*	+*X*	−*a*	−*a*	−*a*	−*a*	+*Z*	−*Z*	−*Z*	−*Z*	−*Z*
NMC = 2, NTC = 10, NSC = 8, TMCC = 320, TTCC = 200, TSCC = 900, TMC = 750, TTC = 265, and TPC = 2435																				

**Table 10:** One of the best process plans for Part 2 under condition (2).

Operation	1	2	18	11	6	12	13	19	17	3	5	7	8	9	10	20	14	4	15	16
Machine	2	2	2	2	2	2	2	2	2	2	2	2	2	2	2	4	4	1	1	1
Tool	7	7	7	7	7	3	9	9	7	7	7	7	3	9	10	10	10	2	1	5
TAD	+*Z*	−*Z*	−*Z*	−*Z*	−*Z*	−*Z*	−*Z*	+*Z*	−*X*	+*X*	+*X*	−*a*	−*a*	−*a*	−*a*	+*Z*	−*Z*	−*Z*	−*Z*	−*Z*
NMC = 2, NSC = 8, TMCC = 320, TSCC = 900, TMC = 750, and TPC = 1970																				

**Table 11:** One of the best process plans for Part 2 under condition (3).

Operation	1	6	2	5	11	12	13	14	18	17	7	8	9	10	19	20	3	4	15	16
Machine	3	3	3	3	3	3	3	3	3	3	3	3	3	3	3	3	3	1	1	1
Tool	6	6	6	6	8	2	9	10	6	8	8	2	9	10	9	10	6	2	1	5
TAD	+*Z*	−*Z*	−*Z*	−*Z*	−*Z*	−*Z*	−*Z*	−*Z*	−*X*	−*X*	−*a*	−*a*	−*a*	−*a*	+*Z*	+*Z*	+*X*	−*Z*	−*Z*	−*Z*
NMC = 1, NSC = 6, TMCC = 160, TSCC = 700, TMC = 1730, and TPC = 2590																				

**Table 12:** Results compared to other algorithms for Part 2.

Condition	Proposed approach	ACO	TS	SA	GA
(1)					
Mean	2456.1	2490.0	2609.6	2668.5	2796.0
Maximum	2527.0	2500.0	2690.0	2829.0	2885.0
Minimum	2435.0	2450.0	2527.0	2535.0	2667.0
(2)					
Mean	2115.4	2117.0	2208.0	2287.0	2370.0
Maximum	2380.0	2120.0	2390.0	2380.0	2580.0
Minimum	1970.0	2090.0	2120.0	2120.0	2220.0
(3)					
Mean	2600	2600.0	2630.0	2630.0	2705.0
Maximum	2740.0	2600.0	2740.0	2740.0	2840.0
Minimum	2580.0	2600.0	2580.0	2590.0	2600.0

## Symbols

*K*: Number of ants
*k*: Index of ant, *k* ∈ [1, *K*]
*u*: Source node
*v*: Destination node
*τ*_*uv*_: Pheromone
*η*_*uv*_: Heuristic information
*α*: Relative weight of pheromone *τ*_*uv*_
*β*: Relative weight of heuristic information *η*_*uv*_
*ρ*: Pheromone evaporation rate
*E*: Algorithm constant to determine *η*_*uv*_
*Q*: Algorithm constant to determine Δ*τ*
*τ*_0_: Initial value of pheromone
PP_*k*_: Process plan achieved by ant *k*
*L*_*k*_: TPC achieved by ant *k*
*S*_*k*_: Set of nodes allowed by ant *k*
PP_*b*_: Up-to-now best process plan
*L*_*b*_: Up-to-now best TPC
PP_*i*_: Iteration best process plan
*L*_*i*_: Iteration best TPC
PP_*r*_: Restart best process plan
*L*_*r*_: Restart best TPC
*L*_avg_: Average value of TPC since the latest restart
*M*_rpt_: Maximum number of repeats
*M*_ite_: Maximum number of iterations
*N*_rpt_: Number of repeats
*N*_ite_: Number of iterations
*R*_ite_: Number of iterations since the latest restart.
